This article has been retracted.

# The Effect of Psychological Support Intervention Based on Structure-Process-Result Three-Dimensional Quality Assessment on Maternal Role Adaptation and Pelvic Floor Rehabilitation Exercise Compliance of Women in Spontaneous Labor

**DOI:** 10.1155/2022/8993144

**Published:** 2022-05-27

**Authors:** Lichun Wang, Lu Shi, Lijun Wang, Yan Wu, Xiaohong Zhang, Tuo Chen, Congmin Huo

**Affiliations:** Department of Obstetrics, Hunan People's Hospital, Changsha, 410000 Hunan, China

## Abstract

**Objective:**

A case-control study was conducted to explore the effect of psychological support intervention based on structure-process-result three-dimensional quality assessment on maternal role adaptation and pelvic floor rehabilitation exercise compliance.

**Methods:**

110 parturients who delivered naturally in our hospital from January 2019 to October 2021 were randomly divided into the control group and the study group. Patients in the former group received routine nursing measures, while patients in the latter group received psychological support intervention based on structure-process-outcome three-dimensional quality assessment (intervention group). Psychological intervention measures include health education, cognitive therapy, behavioral therapy, collective psychological intervention, and happiness therapy. The Edinburgh postpartum depression (PPD) scale and general self-efficacy scale were adopted before intervention, on the day of discharge, and 42 days after delivery. Meanwhile, the mother's role adaptation questionnaire was adopted 42 days after delivery. The PPD, the change of self-efficacy, the function of the pelvic floor, the role adaptation of mothers, and the compliance of pelvic floor rehabilitation exercise in the control group and the intervention group were analyzed.

**Results:**

There was a significant difference in the EPDS score between the two groups at 42 days after delivery. There was a significant difference in the incidence of depression 42 days after delivery between the two groups (*P* < 0.05). The score of pelvic floor function in the two groups after intervention was higher than that before intervention, and that in the intervention group was higher than that in the control group (*P* < 0.05). The score of self-efficacy in the two groups after intervention was higher than that before intervention, and that in the intervention group was higher than that in the control group (*P* < 0.05). The role adaptation of mothers in the intervention group was better than that in the control group (*P* < 0.05). The compliance rate of pelvic floor rehabilitation exercise in the intervention group was higher than that in the control group (*P* < 0.05).

**Conclusion:**

Psychological support intervention based on structure-process-result three-dimensional quality assessment can effectively enhance the sense of self-efficacy, pelvic floor function, maternal role adaptation, and pelvic floor rehabilitation exercise compliance of parturients and can effectively reduce the incidence of PPD and play a positive role in the prevention of PPD.

## 1. Introduction

Postpartum depression (PPD) is one of the common negative emotions of puerperal women [1]. A large number of epidemiological studies have indicated that the prevalence rates of PPD in some countries during the perinatal period are 5%, 30%, and 5%, respectively [1, 2]. All kinds of life, economic, and work pressures they face are increasing, and the incidence of PPD is also increasing year by year [3]. According to the global burden of disease (GBD) statistics in 2010, the worldwide incidence of depression is not low [4]. Depression is expected to jump to second place in 2020, surpassing cancer, cardiovascular and cerebrovascular diseases, and diabetes. The high incidence of PPD will not only affect the physical and mental health of pregnant women but also affect the development of infants and even lead to suicidal or infanticide thoughts or behaviors [5].

Compared with the last generation of parturients, today, most of the parturients have poor self-care ability and strong dependence [6]. The primary parturients lack knowledge of normal pregnancy, childbirth, and parenting without sufficient psychological preparation [7]. The excessive attention of the family members, such as “one-person antenatal examination, accompanied by the whole family,” is also imperceptibly exerting too much pressure on the primary parturients [8]. Therefore, a parturient from pregnancy to parenting has major emotional experiences and physiological changes and is a high-risk group for PPD.

Due to the lack of the development of community nursing, the relevant knowledge needed by parturient women in the perinatal period is difficult to be satisfied [9]. China is now facing the situation that the total nursing human resources are insufficient, which is difficult to meet the physical and psychological needs of pregnant women [9, 10]. Moreover, “patient-centered” high-quality nursing service has been advocated in our country recently [11]. The traditional nursing model is mainly based on nurses' health education and psychological communication with patients. Clinical nursing quality is not only an indispensable part of the overall medical quality but also an important evaluation standard to measure the service quality of medical units [12]. Nursing quality management is to establish the scale of nursing quality according to the process and law of the formation of nursing quality. Scientific nursing decisions are made based on facts and data, so as to meet the needs of service objects and provide patients with safe, efficient, high-quality, and economical nursing services [11, 12]. The purpose of monitoring the nursing quality evaluation index is to improve nursing quality and ensure that patients receive high-quality service.

In 1970, Donabedian first proposed to apply the “structure-process-result” model to the evaluation of medical and nursing service quality. Among them, structure refers to the attributes of the nursing environment, including the manpower, material resources, and financial resources required by nursing services. The process describes the application of structural attributes to practice, that is, all the medical and nursing service processes accepted by patients. The result refers to the final performance brought about by the process, and its purpose is to evaluate whether the nursing program implemented is feasible [10]. Donabedian believed that the structure, process, and results of medical care services were interlinked, influenced each other, and were linearly related.

The three-dimensional quality structure model covers all stages of the nursing clinical care project. The focus of the evaluation is on the basic conditions provided by the hospital for nursing work: (1) organizational structure and staffing: the proportion of bed care structure, the proportion of registered nurses, and the quality of medical staff; (2) the environment and materials of medical institutions: the qualified level of medical devices, instruments, and materials; (3) theoretical knowledge and professional operation level; and (4) management system of the nursing working group: through the formulation of rules and regulations to ensure the effective progress of nursing work, the relevant medical materials are complete, and electronic visibility management is carried out to the maximum extent [11, 12]. At present, it is based on the “structure-process-result” three-dimensional quality evaluation model. In addition, the final quality evaluation of the standard is established by the Delphi method for experts to consult and collate the results. Improving the quality of nursing plays a positive role in maternal role adaptation and pelvic floor rehabilitation exercise compliance. Therefore, through a case-control study, this study focuses on the effect of psychological support intervention on maternal role adaptation and pelvic floor rehabilitation exercise compliance.

## 2. Patients and Methods

### 2.1. General Information

A total of 110 women with spontaneous delivery and parturition treated in our hospital from January 2019 to October 2021 were randomly assigned into the control group and the intervention group. Patients in the control group received routine nursing measures, while patients in the study group received psychological support intervention based on structure-process-result three-dimensional quality evaluation (intervention group). The age of the control group was 20-33 years, with an average of 26.45 ± 2.81 years, and that of the intervention group was 20-34 years, with an average of 26.57 ± 3.31 years. There exhibited no statistical significance in the general data. This study was permitted by the Medical Ethics Association of our hospital, and all patients signed informed consent.

*Inclusion criteria*: (1) first parturient women have singleton pregnancy whose gestational weeks are 28-42 weeks and age is 20-35 years; (2) pregnant women and their families have a certain understanding, language expression, and writing skills; (3) pregnant women and their families voluntarily participate in the study and sign the informed consent form and follow the random principle; and (4) the first pregnant women and their families will use mobile Wechat, QQ, and other network tools.

*Exclusion criteria*: (1) patients with a history of mental illness or family mental illness or receiving related treatment; (2) severe organ diseases; (3) chronic diseases during or before pregnancy, such as chronic hypertension, chronic pulmonary disease, heart disease, diabetes, and hepatorenal disease; (4) preterm or postoperative complications, such as postpartum hemorrhage, uterine rupture, and amniotic fluid embolism; and (5) experience of major stress events in recent months.

### 2.2. Treatment Methods

The control group was given routine nursing, including (1) maternal and infant symptoms, medication management, psychological nursing, and rehabilitation diet and exercise education before and after delivery in the hospital; (2) routine nursing of newborns, including breastfeeding, neonatal bathing, touching, skin, buttocks, and navel care, neonatal stress reaction, complexion, and defecation observation to judge whether the baby is cold or warm; (3) health education. The methods of health education include face-to-face education, handbook distribution, and department publicity; (4) guidance before discharge; and (5) 42 days after delivery, researchers remind parturients to come to the hospital for health check-ups.

The patients in the intervention group received psychological support intervention based on three-dimensional quality management based on “structure-process-results.” Meanwhile, the Delphi method was applied to consult the experts and organize consultation results. The specific methods are as follows: (1) a research group was set up consisting of two senior obstetrics and gynecology experts, one head nurse in obstetrics and gynecology, and eight specialist nurses. The intervention group revolves around three-dimensional quality management and compiles the postpartum nursing quality evaluation standard system by the method of literature retrieval. The intervention group includes work characteristics, key links, and quality control; (2) experts with at least 10 years' experience in obstetrics and gynecology in the province and city were selected as letters to consult the experts, and the intervention group was finally invited to consult the experts in the intervention group. The contents of the letter table were evaluated by the letter inquiry experts through the Delphi method according to the Likert intervention group score method. All the letter inquiry experts expressed their opinions anonymously and were not allowed to communicate with each other. The specialist nurses of the intervention group recorded and sorted out the evaluation of the contents of the letter table by the letter inquiry experts; (3) the specialist nurses will sort out the results of the first round of evaluation to the group for discussion, select the items with different opinions to compile the second letter table, and invite the experts again to use the Delphi method to evaluate them. After the letter inquiry, the items at all levels are integrated according to the expert opinions and the weight coefficients of each evaluation index, to form a nursing quality evaluation system for women with natural labor and first birth. The responsible nurses are led by the head nurse to learn and give different nursing tasks to nurses with different nursing experiences, which can be applied to clinical nursing; and (4) psychological intervention. When the patient is hospitalized, the nursing staff should record the patient's personal information in detail and have a general understanding of the patient's psychological situation and personality characteristics. When carrying out psychological intervention for patients, psychological counseling should be carried out according to the psychological state of patients and the specific degree of cognition. Establish a trusting communication relationship with the patients, understand the psychological changes, and choose the appropriate way of communication and language expression according to the patients' educational background. In the whole process of nursing, patients should be respected and encouraged and given warmth. For some patients with more prominent psychological problems or special conditions, professional psychological counseling should be carried out, patients should be guided to vent in time, and psychotherapeutic measures should be implemented. Each patient is given a self-made “health manual” on postpartum care, which can be presented in cartoons to improve patient acceptance, taking into account the patient's emotional status. It should be noted that the formulation of the health manual should be concise and easy to understand as far as possible to avoid the psychological burden of too long space on patients. Finally, the knowledge of diet and daily rest and activities should be emphasized to provide all-round care for patients. The patient received 20 min education 3 times a week after admission. Cognitive therapy: first parturient women will have varying degrees of psychological problems after delivery, mostly anxiety and depression, and then will treat and deal with everything passively. Therefore, nurses should correct patients' wrong cognition in time, pay attention to communication skills in this process, and avoid pointing out their mistakes too bluntly, so as not to cause resistance and extreme behavior. The steps to change the wrong thinking of pregnant women are as follows: (1) first, listen to their views on people and things, understand their inner feelings, and understand their thinking and behavior as much as possible; (2) do not evaluate their subjective views and guide patients to evaluate themselves objectively; (3) use positive cases to help pregnant women strengthen their confidence, improve their courage to face problems, and get rid of pessimism; (4) provide parturients with some specific coping strategies, such as going out to play and listening to music. Collective psychological intervention: the psychological intervention collective consists of psychological counseling, an obstetrician and gynecologist, a nurse, and a pregnant woman receiving psychological intervention. All members do not change groups or withdraw at will during the period of psychological intervention. Collective is an economical and effective method, which has become the consensus of professional helpers. In groups of no more than 10 people, the training is mainly conducted by psychological counselors; there will be 42 days of postpartum reexamination after discharge in our hospital, which can be carried out during the treatment of pelvic floor rehabilitation, a total of 10 times, 2-3 times per week, lasting for one month, 40 min in each group. Starting from the establishment of a relationship of mutual trust, ask questions when pregnant women are open, provide feedback during description and role-playing in psychological dramas, and guide them to slowly adapt to the role of mothers and face life positively and optimistically. Attitudes and behaviors learned in groups, that is, changed emotions and cognition, are more likely to migrate to real life. Happiness therapy: for pregnant women with a stable condition and good control of complications, nurses and their families should help patients learn physical and mental self-management. Master the personality characteristics, work style, and psychological characteristics of the patients, give appropriate nursing, inform the patients that the postpartum symptoms are normal, and give sympathy, support, and encouragement. Correct the negative thoughts of pregnant women and work with them to explore the negative effects of negative perceptions and misunderstandings on the body and mind in order to reduce anxiety and depression.

### 2.3. Observation Index

On the day of discharge, the paper questionnaire was distributed on the spot or the data were collected through the Internet link. The questionnaire included three questionnaires: general condition questionnaire of parturient, Edinburgh PPD scale (EPDS) [11], and general self-efficacy scale (GSES) [12]. About 42 days after delivery, the first parturient filled out three questionnaires: EPDS, GSES, and maternal role adaptation questionnaire. Those with EPDS ≥ 10 were classified as depression, and those with EPDS < 10 as nondepression. Pelvic floor function: the Phenix pelvic floor functional rehabilitation exercise system was used to evaluate the muscle strength of type I and II muscle fibers of the pelvic floor. If the subjects are unable to use the Internet, the researchers will call to ask for their options and fill in them instead or during the 42-day postpartum health check-up of the parturient, comparing maternal role adaptation and pelvic floor rehabilitation exercise compliance after the intervention. The pelvic floor muscle exercise compliance scale was used to evaluate the pelvic floor muscle exercise compliance of the two groups before and after the intervention, including time, action standardization, and other contents; the total score was 100 points, more than 90 points as complete compliance; 60-90 points as incomplete compliance; less than 60 points as complete noncompliance; complete compliance and incomplete compliance were generally counted as the total compliance rate. After the preexperiment, consistency reliability Cronbach's *α* and validity coefficient of the questionnaire were 0.91 and 0.80, respectively.

### 2.4. Statistical Analysis

All the data in the study were analyzed by the Chinese version of the intervention group SPSS22.0 intervention group statistical software, with the intervention group *P* < 0.05. There was statistical significance in the intervention group. The counting data of general data are presented by frequency and percentage, the measurement data are described by the mean ± standard deviation, and the correlation between parturient's self-efficacy and prenatal depression is analyzed. The balance test of the general data of parturients was analyzed by two independent sample intervention group *t* test and chi-squared test. The changes in PPD and self-efficacy of parturients in the comparison group were evaluated by repeated measurement analysis of variance; the scores of PPD, self-efficacy, maternal role adaptation, and pelvic floor rehabilitation exercise compliance were compared by the *t* intervention group test and chi-squared test, and the intervention effect was evaluated.

## 3. Results

### 3.1. Comparison of the Balance of Basic Data of Research Objects

First of all, we compared the balance of the basic data of the subjects. There were 110 subjects, 55 in the control group and 55 in the intervention group. The average age of the control group was 26.45 ± 2.81 years (20-33 years). The average age of the intervention group was 26.57 ± 3.31 years (20-34 years). By *t* test, *P* > 0.05, the difference exhibited not statistically significant. And there was no significant difference in different ages, only child, education, occupation, family income, planned pregnancy, sex expectation of baby, relationship between husband and wife and mother-in-law, sleep quality, and feeding mode (*P* > 0.05). All the results are indicated in Table 1.

### 3.2. Comparison of EPDS Scores before Delivery, on the Day of Discharge, and 42 Days after Delivery between the Control Group and the Intervention Group

We compared the EPDS scores before, on the day of discharge, and 42 days after delivery. On the day of admission, the prenatal EPDS scores ranged from 1 to 18. By the independent sample *t* test, there exhibited no significant difference in EPDS scores on the day of admission (*P* > 0.05); on the day of discharge, there exhibited no significant difference in EPDS scores (*P* > 0.05); there exhibited a significant difference in the score of EPDS at 42 days postpartum (*P* < 0.05). All the results are indicated in Table 2.

### 3.3. Comparison of the Incidence of Depression before, on the Day of Discharge, and 42 Days after Delivery between the Two Groups

We compared the incidence of depression before, on the day of discharge, and 42 days after delivery. The incidence of depression was 23.64% and 21.82%, respectively. By the chi-squared test, there exhibited no significant difference in the incidence of prenatal depression (*P* > 0.05). On the day of discharge, there exhibited no significant difference in the incidence of depression (*P* > 0.05), but there exhibited a significant difference in the incidence of depression 42 days after delivery (*P* < 0.05). All the results are indicated in Table 3.

### 3.4. Comparison of Pelvic Floor Function between the Two Groups

We compared the pelvic floor function, and there exhibited no significant difference in the scores of pelvic floor function before intervention (*P* > 0.05). The score of pelvic floor function after intervention was higher compared to that before intervention, and the score in the intervention group was higher compared to the control group (*P* < 0.05). All the results are indicated in Table 4.

### 3.5. Comparison of Self-Efficacy Scores between the Two Groups

We compared the scores of self-efficacy (skills, inner activity, and breastfeeding), and there exhibited no significant difference in the scores of self-efficacy before intervention (*P* > 0.05). The scores of self-efficacy after intervention were higher compared to that before intervention, and the scores in the intervention group were higher compared to the control group. All the results are indicated in Table 5.

### 3.6. Comparison of Maternal Role Adaptation between the Two Groups

We compared the maternal role adaptation: the maternal role adaptation after intervention in the intervention group was good in 16 cases, moderate in 37 cases, and poor in 2 cases, while in the control group, the maternal role adaptation was good in 6 cases, moderate in 20 cases, and poor in 29 cases. The maternal role adaptation of the intervention group was better compared to that of the control group (*P* < 0.05). The specific results are indicated in Figure 1.

### 3.7. Comparison of Compliance of Pelvic Floor Rehabilitation Exercise between Two Groups

We compared the compliance of pelvic floor rehabilitation exercise. In the intervention group, there were 34 cases of complete compliance, 17 cases of incomplete compliance, and 4 cases of complete noncompliance, with a compliance rate of 92.73%, while the control group had complete compliance in 20 cases, incomplete compliance in 19 cases, and complete noncompliance in 16 cases, with a compliance rate of 70.91%. The compliance rate of patients in the intervention group was significantly higher compared to that of the control group (*P* < 0.05). The compliance rate of pelvic floor rehabilitation exercise in the intervention group was significantly higher compared to that of the control group (*P* < 0.05). The specific results are indicated in Figure 2.

## 4. Discussion

The primary parturients lack knowledge of normal pregnancy with sufficient psychological preparation [7]. Therefore, pregnant women who usually experience various physiological changes will become a high-risk group for postpartum depression [12].

Postpartum depression includes a group of emotional disorders. The “baby blues” usually peak in the first five days after delivery and tend to recover quickly [13]. Severe postpartum depression is a disease that meets the clinical diagnostic criteria of depression and needs targeted drug treatment and psychotherapy. We do know that a personal history of a mood illness or anxiety, particularly if present and untreated throughout pregnancy, is the best predictor of postpartum depression. Women who have a history of depression during pregnancy are seven times more likely to suffer from major postpartum depression [14].

Hospital nurses combined with the actual situation of parturients take appropriate health knowledge guidance and can also significantly promote the quality of life and the level of physical and mental health of parturients, which is conducive to the healthy growth of newborns [15]. The research on PPD is mainly focused on how to evaluate the diagnosis of PPD and evaluate the high-risk factors of depression and timely prevention intervention methods.

At present, the intervention research on PPD is mainly through early screening, early detection and early intervention, early psychological counseling, health education, and the establishment of a reasonable health education system [16]. Some intervention studies are mostly carried out during the hospitalization of pregnant women, that is, before and after delivery. In some countries, the intervention during maternal hospitalization is more important than in the community. Several surveys have indicated that screening of prenatal depression can help to identify and treat PPD effectively with consistent results of the Radoš et al. study [17]. Positive psychological assessment and intervention are able to effectively prevent or reduce PPD [18]. Nakamura et al. believe that the correct implementation of a maternal mental health education program can obviously relieve the symptoms of PPD via strengthening social support and increasing self-efficacy [19]. At present, the research on PPD in China is still in the preliminary stage; few studies have been reported till now. Our research filled in some of the gaps in PPD.

Our results indicated that there exhibited a significant difference in the EPDS score at 42 days postpartum (*P* < 0.05). About 42 days after delivery, the incidence of depression was statistically significant. The pelvic floor function scores of the two groups after intervention were higher than those before intervention, and the score of pelvic floor function in the intervention group was higher compared to that of the control group. The score of self-efficacy after intervention was higher compared to those before intervention, and the score in the intervention group was higher compared to that in the control group. The maternal role adaptation of the intervention group was better compared to that of the control group. The compliance rate of patients in the intervention group was significantly higher compared to that of the control group, and the compliance rate of pelvic floor rehabilitation exercise in the intervention group was higher compared to the control group. According to the analysis of the reasons, the intervention group was given psychological support intervention based on structure-process-result three-dimensional quality evaluation, and nurses paid attention to the changes in the maternal physical and mental state before and after delivery [20–22]. Through nurse-patient communication and health education to guide the new mothers to actively participate in neonatal nursing, we inspire pregnant women to actively learn, produce self-cognition and self-affirmation in practice, and promote interaction and support among parturients, spouses, and family members. Through psychological nursing intervention, parturients can observe, learn, and experience the role of novice mothers in nursing work, realize the problems caused by their negative emotions, and directly adjust their physical and mental state with the help of family members and nurses [23, 24]. It is helpful to relieve maternal anxiety, relax the body and mind, reduce loneliness, change maternal physical and mental quality, and enhance satisfaction.

Conclusively, psychological support intervention based on structure-process-result three-dimensional quality assessment can effectively control the incidence of PPD and play a positive role in the effective prevention of PPD. The psychological support intervention based on structure-process-result three-dimensional quality assessment can help primary parturients to participate in taking care of their babies more confidently, effectively promote their sense of self-efficacy, and then effectively enhance their family harmony, the maternal role adaptation, treatment compliance, and pelvic floor rehabilitation compliance of parturient women.

## Figures and Tables

**Figure 1:** Comparison of maternal role adaptation between the two groups.

**Figure 2:** Comparison of compliance to pelvic floor rehabilitation exercise between the two groups.

**Table 1:** Comparison of general equilibrium between the control group and the intervention group (%).

Related factors	Control group (*n* = 55)		Intervention group (*n* = 55)		*χ* ^2^	*P*
	*N*	Percentage of people	*N*	Percentage of people		
Age (years)					0.570	>0.05
20~25	18	32.73%	19	34.55%		
26~30	33	60.00%	30	54.55%		
31~35	4	7.27%	6	10.91%		

Education level of parturient women					2.324	>0.05
Junior high school and below	10	18.18%	7	12.73%		
High school or technical secondary school	13	23.64%	18	32.73%		
Junior college or bachelor degree	30	54.55%	30	54.55%		
Master's degree or above	1	1.82%	0	0.00%		

Occupation of parturient women					1.425	>0.05
Be unemployed	10	18.18%	9	16.36%		
Farmers	6	10.91%	3	5.45%		
Civil servants	18	32.73%	17	30.91%		
Corporate profession or freelance	21	38.18%	25	45.45%		

The literacy of the spouse					1.230	>0.05
Junior high school and below	6	10.91%	9	16.36%		
High school or technical secondary school	15	27.27%	11	20.00%		
Junior college or bachelor degree	34	61.82%	33	60.00%		
Master's degree or above	1	1.82%	1	1.82%		

Spouse occupation					1.007	>0.05
Be unemployed	2	3.64%	3	5.45%		
Farmers	8	14.55%	7	12.73%		
Civil servants	20	36.36%	16	29.09%		
Corporate profession or freelance	25	45.45%	29	52.73%		

Monthly household income (yuan)					1.992	>0.05
<2000	3	5.45%	6	10.91%		
2000~4000	22	40.00%	17	30.91%		
4000~6000	18	32.73%	18	32.73%		
>6000	11	20.00%	14	25.45%		

Do you have a history of bad pregnancy?					0.573	>0.05
Yes	44	80.00%	47	85.45%		
No	11	20.00%	8	14.55%		

Is this pregnancy part of the plan?					3.117	>0.05
Yes	42	76.36%	49	89.09%		
No	13	23.64%	6	10.91%		

Do you have any expectations for baby sex?					0.227	>0.05
None	45	81.82%	43	78.19%		
Yes	10	18.18%	12	21.82%		

Marriage relationship					0.210	>0.05
Yes	53	96.36%	52	94.55%		
Make do with	2	3.64%	3	5.45%		
Divorce	0	0.00%	0	0.00%		

Sleep quality of parturients in the last week					1.902	>0.05
Fine	7	12.73%	5	9.09%		
Better	21	38.18%	16	29.09%		
Poor	20	36.36%	24	43.64%		
Very bad	7	12.73%	10	18.18%		

Baby feeding mode					1.140	>0.05
Breastfeeding	35	63.64%	34	61.82%		
Artificial feeding	3	5.45%	6	10.91%		
Mixed feeding	17	30.91%	15	27.27%		

The health status of the baby					1.090	>0.05
Normal	52	94.55%	49	89.09%		
Abnormal	3	5.45%	6	10.91%		

**Table 2:** Comparison of EPDS scores before delivery, on the day of discharge, and 42 days after delivery between the control group and the intervention group ($\bar{x}\pm s$, points).

Group	*N*	On the day of admission	On the day of discharge	42 days after delivery
Control group	55	9.37 ± 3.68	9.83 ± 3.41	9.87 ± 4.07
Intervention group	55	9.76 ± 3.73	8.56 ± 3.39	7.25 ± 3.36
*t*		0.552	1.959	3.682
*P*		>0.05	>0.05	<0.01

**Table 3:** Comparison of the incidence of depression before delivery, on the day of discharge, and 42 days after delivery between the control group and the intervention group (*n*, %).

Group	*N*	On the day of admission		On the day of discharge		42 days after delivery	
		Depression	No depression	Depression	No depression	Depression	No depression
Control group	55	13 (23.64)	42 (76.36)	13 (23.64)	42 (76.36)	15 (27.27)	40 (72.73)
Intervention group	55	12 (21.82)	43 (78.18)	9 (16.36)	46 (83.64)	5 (9.09)	50 (90.91)
*χ* ^2^		0.052		0.909		6.111	
*P*		>0.05		>0.05		<0.05	

**Table 4:** Comparison of pelvic floor function between the two groups ($\bar{x}\pm s$).

Group	*N*	Pelvic floor type I		Pelvic floor type II	
		Before intervention	After intervention	Before intervention	After intervention
Control group	55	1.35 ± 0.53	2.21 ± 1.43^a^	1.33 ± 0.64	2.18 ± 1.13^a^
Intervention group	55	1.34 ± 0.26	3.62 ± 1.04^b^	1.27 ± 0.56	3.34 ± 0.85^b^
*t*		0.127	5.914	0.523	6.084
*P*		>0.05	<0.01	>>0.05	<0.01

Note: comparison between the two groups before and after treatment, ^a^*P* < 0.05; comparison between the two groups before and after treatment, ^b^*P* < 0.05.

**Table 5:** Comparison of self-efficacy scores (skills, inner activity, and breastfeeding) between the two groups ($\bar{x}\pm s$).

Group	*N*	Skills	Inner activity		Breastfeeding		
		Before intervention	After intervention	Before intervention	After intervention	Before intervention	After intervention
Control group	55	23.82 ± 2.27	26.98 ± 4.26^a^	25.63 ± 3.51	29.42 ± 2.48^a^	23.13 ± 4.94	27.78 ± 3.46^a^
Intervention group	55	24.11 ± 3.13	36.84 ± 3.42^b^	25.29 ± 4.43	34.56 ± 3.48^b^	22.86 ± 5.25	35.51 ± 4.42^b^
*t*		0.556	13.385	0.446	8.920	0.278	10.213
*P*		>0.05	<0.01	>0.05	<0.01	>0.05	<0.01

Note: comparison between the two groups before and after treatment, ^a^*P* < 0.05; comparison between the two groups before and after treatment, ^b^*P* < 0.05.

## Data Availability

No data were used to support this study.
